# Influence of the Integrated Delivery System on the Medical Serviceability of Primary Hospitals

**DOI:** 10.1155/2021/9950163

**Published:** 2021-08-02

**Authors:** Wenming Feng, Xin Feng, Ping Shen, Zhen Wang, Bing Wang, Jiantong Shen, Xuhui Shen

**Affiliations:** ^1^Department of Medicine, Huzhou University, Huzhou, Zhejiang, China; ^2^University of Sydney, Sydney, Australia; ^3^Zhili Health Center, Huzhou, Zhejiang, China

## Abstract

**Objective:**

To explore the change in the medical serviceability of primary hospitals since the establishment of the Huzhou No. 1 People's Hospital medical care group incorporating the integrated delivery system.

**Methods:**

With reference to the “Grade Evaluation Standard of General Hospitals in Zhejiang Province” and the “Guidelines for Service Capacity Evaluation of Township Hospitals (2019 Edition),” we analyzed the influence of the integrated delivery system on the capacity of primary medical services and selected the targeted core indicators. From the four dimensions of diagnosis and treatment breadth, diagnosis and treatment efficiency, surgical ability, and patient satisfaction, an index evaluation system was established to explore the changes in the medical serviceability in primary hospitals.

**Results:**

The measurements were aimed at four specific issues, that is, the low medical technology level of grassroots personnel, the poor information communication among medical institutions, the difficulty in recruiting people, and the imperfect training mechanism in primary hospitals. After establishing a series of measurements related to the problems faced by the primary healthcare sector in China, the score of breadth of diagnosis and treatment, efficiency of diagnosis and treatment ability, surgical ability, and patient satisfaction of the primary hospitals in our medical group have greatly increased.

**Conclusion:**

The integrated delivery system improved the primary hospitals' medical health ability obviously. Our study also provides various useful and operable suggestions for primary healthcare.

## 1. Introduction

With the rapid development of industrialization and urbanization and the increasingly aging population, the health field is facing challenges related to various infectious and chronic diseases as well as numerous other major public health safety issues. WHO proposed that the integrated delivery system is the most appropriate method for addressing the emerging global health problems. In fact, WHO officially describe integrated health services as a system wherein “continuous services such as health promotion, disease prevention, diagnosis, treatment, disease management, rehabilitation, and nursing treatment are provided according to the needs of different stages of the lifecycle of the population through the cooperation between different levels of medical institutions in the health system” [1]. For certain, the development of a more integrated, people-centered care system has the potential to bring significant benefits to our health and the provision of healthcare for all, including improved access to care, enhanced ownership and clinical outcomes, improved health literacy and self-care, increased satisfaction with care services, increased job satisfaction among healthcare workers, improved service efficiency, and an overall cost reduction [2–4].

In December 2016, the National Health and Family Planning Commission in China further promoted the construction of a medical consortium and proposed the establishment of a guiding mechanism with consistent responsibilities and rights aimed at ensuring that the medical association becomes a community of service, responsibility, benefit, and management, one that effectively allows sharing the medical resources in the region and further improving the grassroots service capacity [5]. Here, it is crucial to promote the formation of a hierarchical diagnosis and treatment mode of community hospitals' primary diagnosis, two-way referral, separate rapid and slow treatment, and linkage between the upper and lower levels. Without the health of the population as a whole, there will exist no comprehensively well-off society. The foundation of national health lies at the grassroots level. China's primary healthcare sector covers a wide range of health facilities, including community health centers and community health stations in urban areas, township health centers, and village clinics in rural areas [6]. In recent years, the governmental bodies at all levels have taken a series of measures to strengthen the construction of primary medical institutions and have achieved relatively positive results.

However, due to various reasons, the weak service capacity of primary medical institutions remains unsatisfactory. Previous studies have found that China's primary health system is facing great challenges, including the insufficient education and qualification of the labor force [7]; poor quality of care [8]; the fragmentation of the health information technology system [9]; and a lack of digital data, insurance policies that hinder nursing efficiency, and poor control performance of the risk factors. Meanwhile, a number of overseas studies have directly examined the impact of medical alliances on primary medical and health institutions, largely in terms of the evaluation of the effect and performance of integrated health services, including the evaluation of the quality of primary healthcare [10]. The present study is aimed at quantitatively evaluating the influence of the integrated delivery system on the medical serviceability of primary hospitals and identifying an effective way to improve the primary healthcare in China's hospitals.

## 2. Huzhou No. 1 Hospital Model

### 2.1. Background

The Huzhou No. 1 People's Hospital medical care group was established in March 2019. Led by the Huzhou First People's Hospital (tertiary general hospital), the member units include Wuxing hospital district (secondary general hospital), as well as Daixi, Balidian, Donglin, Zhili, Daochang, and Miaoxi hospitals, which form a “1 + 1 + 6” three-level urban medical community model of one municipal general hospital, one district general hospital, and six township health centers (including 63 stations). Unlike the county medical community model, the “1 + 1 + 6” three-level urban medical community model has the characteristics of a cross-urban two-level government, with a wide geographical distribution, and an uneven level scale. In view of these characteristics, the group has constructed a continuous medical service system of a “direct line covering the whole area and providing a continuous service” in cities, districts, and towns; has built a model area for the construction of a national urban medical community as part of the group's vision; and has gradually promoted the construction of an urban medical community.

### 2.2. Index Evaluation System

We used the fishbone analysis method to analyze our system.  Figure 1 shows the procedure of our analysis of the issues faced by the primary hospitals in our integrated group. Following voting by the committee, the main factors were selected.

With reference to the “Grade Evaluation Standard Of General Hospitals in Zhejiang Province” and the “Guidelines for Service Capacity Evaluation of Township Hospitals (2019 Edition),” the core indicators affecting the primary medical service capacity were screened and the index evaluation system was established as follows:

1. The breadth of diagnosis and treatment: the number of diagnosis-related groups (DRGs) in secondary hospitals, the number of township health centers along with the number of outpatient outcomes achieving the standard, and the coverage rate of family doctors assigned by the key groups
2. The efficiency of diagnosis and treatment: the average number of doctors per day, the utilization rate of beds, and the average length of stay
3. Surgical ability: the proportion of operations above grade II (all kinds of operations with high technical difficulty, complicated operation process, and high risk), the operations carried out, and the types of therapeutic operation
4. Patient satisfaction: inpatient satisfaction and outpatient satisfaction

### 2.3. Problem and Solutions

Through the voting of various quality management team members, the real reasons for the low serviceability of primary hospitals were obtained. The following sections address the root causes and the measurements related to improving the primary healthcare in our hospital.

### 2.4. The Poor Medical Technology Level of Grassroots Personnel

With the improvement of the economic level and the increase in the incidence of chronic diseases, the staff's ability to use the medical technology in primary hospitals is not sufficient for handling the increasing health needs. Moreover, more and more patients are seeking care from community health centers or township hospitals since they have little trust in the knowledge or skills of their family doctor [11]. In accordance with the characteristics of each hospital and each district, we must address the directional delegation of medical talents and the hierarchical guidance and must improve the technical level.

In terms of the chronic diseases within the group, we built a matrix management platform based on the integrated delivery system. Through the improvement of the hierarchical diagnosis and treatment system, the management of chronic diseases was assigned to the grassroots community, with family doctors responsible for the disease management of patients with chronic diseases. At the same time, relevant experts were encouraged to join the family doctor team and provide medical services to improve the quality of the primary medical services. The unique attitude, skills, and knowledge of family doctors qualify them to provide continuous and comprehensive healthcare and prevention services to each family member [12]. Moreover, a party-building alliance was set up and the medical backbone team and member units were sent to assist in terms of one-on-one consultations. Meanwhile, we also formulated an accurate teaching plan to improve the medical level of the grassroots personnel.

### 2.5. Poor Information Communication among Medical Institutions

The lack of information communication among medical institutions is a major issue for the integrated medical group. In the construction of the integrated delivery system, the development of “internet-based medical health” and the promotion of telemedicine are the key factors. Here, we built a long-distance consultation and two-way referral system (Figure 2), strengthened the information communication, and built a “first-line direct” continuous medical service system, covering the whole area and providing a continuous service.

The rapid development of cloud computing, mobile health applications, Big Data, and the Internet of Things could help to optimize the medical process and improve service efficiency, which is indispensable to promoting the profound transformation of medical services and management modes [13]. Here, teleconsultation is used to address three broad challenges in the delivery of care: geographical barriers, logistical barriers, and lack of specialist support [14]. We used a 5G network for the remote consultation of grassroots patients, ensuring it was more convenient to access a doctor. By using cloud classrooms, the general hospital can connect multiple branches to carry out remote live broadcasts and teaching at the same time, such that the innovative medical information can be efficiently communicated through the integrated medical group. We opened a number of referral channels for patients who meet the specific criteria through a hierarchical diagnosis and treatment information system. This system presents an effective way to make full use of the limited medical resources and to treat more patients with chronic diseases by establishing a hierarchical diagnosis and treatment system while dividing the patients presenting different conditions into different levels of the hospital.

### 2.6. Difficulty in Recruiting People in Primary Medical Institutions

The lack of high-quality talents leads to a weak technological basis and an unreasonable structure of talent, which results in being unable to meet the developmental needs of primary medical and health services as well as the needs of the grassroots people. When compared with hospitals, there is a clear lack in the working environment of primary medical and health institutions. Low wages, poor employment environments, and fewer opportunities for promotion and training are the main factors behind the primary medical institutions' inability to retain health talents. In short, there is a global shortage of skilled practitioners, while China specifically needs to develop a talent pool to support its ambitious primary healthcare reform agenda [15]. To resolve this issue, it is important that all internal members are recruited in a unified way to ensure the needs of the grassroots personnel.

We unified the legal position of each member unit and built 14 centers (see Figure 3) to standardize hospital recruitment standards and to allocate recruitment tasks in a reasonable manner. A unified recruitment plan should be formulated within the scope of the total number of grassroots posts and the proportion within the overall structure, with the leadership of the medical community organizing the unified recruitment, reflecting the principle of who is in charge and who is responsible. After the recruitment results have been determined, the county-level hospitals will uniformly assign and set the various posts. In accordance with the needs of the primary medical services, the geographical distribution of primary medical and health institutions must be addressed, the comprehensive quality of the potential personnel must be guaranteed, the distribution direction must be determined, and a tripartite employment contract must be signed to enhance the pertinence of recruitment work. Meanwhile, for the medical students who are about to graduate, comprehensive administrative measures must be formulated to ensure that they abide by the contract related to serving rural health enterprises following graduation. To a certain extent, these methods will effectively resolve the shortage of grassroots medical staff and the difficulties in recruitment.

### 2.7. The Imperfect Training Mechanism of Primary Medical Institutions

With the rapid development of medical technology, new technologies and new knowledge are constantly emerging. Only through reasonable and effective training, the timely updating of professional knowledge, and an improvement in the quality level can we meet the requirements of society. The backwardness in the area of training has led to the issues of poor medical quality, difficult doctor-patient relationships, an increasing number of contradictions, hospital management confusion, and “brain drain.” It is thus crucial to unify the training for all members of the group to improve the ability of the grassroots personnel.

The training programs need to identify the capabilities required to meet the health needs and priorities of the local community within the context of a multidisciplinary team, rather than simply copying ideas and courses from a richer resource context [16]. This could be achieved through distance teaching, improving the level of primary medical care, and building a specific capacity training center. For example, secondary and tertiary hospitals could provide professional guidance to grassroots doctors through live lectures, online learning, and establishing a professional knowledge base, such that the patients are better served. Here, we requested that the training content, the lecturer, the organizer, the training assessor, and the evaluation standard are clarified. At the same time, we clarified the knowledge and skills that different posts and different levels of personnel need to master, combining this with the actual situation of the hospital to formulate a unified and scientific training curriculum system.

### 2.8. Performance of Healthcare Services

Table 1 shows the performance of the healthcare units in Huzhou No. 1 People's Hospital before and after taking the measures. In accordance with the scoring criteria, we obtained the score for each subject in relation to four dimensions. The total score was increased from 64 to 87 after we implemented certain measures in the primary healthcare units. It is clear that the integrated delivery system has had a positive effect on the number of DRG groups in secondary hospitals and the standard rate of the number of outpatients in township hospitals. In addition, the contracted coverage rate of family doctors, the average daily diagnosis and treatment times of doctors, the bed utilization rate, the types of operation and the therapeutic operations in township hospitals, and the level of satisfaction in outpatient and inpatients departments are all increasing.

## 3. Discussion

With the acceleration of urbanization and the increasingly aging population, the burden related to chronic diseases and the brain drain of health professionals in rural areas are becoming increasingly serious issues. This has expanded both the demand and the scope of the primary healthcare sector, thus increasing the demand for qualified primary healthcare workers [17]. The weak grassroots level presents a major limitation that has long restricted the high-quality development of health services, and it is also the greatest hindrance to the construction of an integrated medical and health service system. At present, China's primary healthcare is facing challenges: the suboptimal education and training of primary healthcare practitioners, a fee-for-service payment system that incentivises testing and treatments over prevention, fragmentation of clinical care and public health service, and insufficient continuity of care throughout the entire healthcare system [18]. The difficulty in intensifying the reform of the medical system lies at the grassroots level, while this level continues to remain the main source of vitality. Therefore, it is important to promote the restructuring of county medical and health resources, to undertake a system reconstruction, a mechanism reconstruction, and a service remodeling, as well as realizing the upgrading of grassroots serviceability, which will mark the breakthrough of the reform. The construction of the county medical community is an important factor for exploration and any breakthrough here could help resolve the issues in the primary medical system. Here, the key is to establish a new medical and health service system and a revolutionary reform in the field of health [19].

The construction of the integrated delivery system is an effective means for realizing hierarchical diagnosis and treatment patterns as well as an important means for improving the quality and efficiency of China's medical service supply system. The upper and lower medical institutions within the medical association should establish a division of labor and various cooperation mechanisms while clarifying the rights, responsibilities, and interests of all parties, enhancing the channels for resource circulation, and improving the serviceability of lower-level medical institutions. The medical alliance provides the possibility of clarifying the management system and the operation mechanism of the division of labor and enhancing the cooperation among the different levels within the medical institutions. It also allows for the integration of the scattered institutions developed by the original monomer into a community of strategy, interest, responsibility, and management, providing the driving force for reversing the plummeting high-quality medical resources. The alliance also presents a powerful starting point for promoting the construction of a hierarchical diagnosis and treatment system, while it is also the key to controlling medical expenses and enhancing the satisfaction of the people we serve [20].

Although the existing research has explored the application of the integrated medical system, the evaluation of the integrated medical system was still a lack of systematic indicators. To promote the primary care capacity in our medical group, we first created an index evaluation system. With reference to the “Grade Evaluation Index of General Hospitals in Zhejiang Province” and the “Guidelines for Service Capacity Evaluation of Township Hospitals (2019 Edition),” the core indicators affecting the primary medical service capacity were screened and selected by the committee. The indicators were divided into four dimensions: the breadth of diagnosis and treatment, the efficiency of diagnosis and treatment ability, surgical ability, and patient satisfaction.

In terms of the specific methods, we proposed various measurements based on the local conditions. The medical personnel should be directed and guided at different levels according to the characteristics of each hospital and each district. It is important to build a remote consultation and two-way referral system to strengthen information communication. Moreover, internal members should be recruited in a unified manner to ensure the needs of the grassroots personnel are met. In addition, a unified, rigorous, and practical training and evaluation system should be established to promote the development of the community health service system in mainland China [21]. The results of the evaluation of the primary healthcare capacity before and after the measures were implemented allowed us to ascertain the effect of the integrated delivery system on primary healthcare. In short, the integrated delivery system has had the greatest impact on increasing the breadth of diagnosis and treatment, while the other dimensions were all found to be slightly improving.

This study involved certain limitations. First, since Huzhou is a small city in China, the attendant healthcare ability does not represent the ability of China as a whole, which means it is important to perform further appropriate measurements according to the local conditions. Moreover, with the rapid development of living standards and the increasing demands for medical services, the evaluation criteria in our system will perhaps no longer apply to the future medical needs. Therefore, the evaluation system for grassroots serviceability needs to be further improved. In the hierarchical diagnosis and treatment system, the diagnosis of a patient's condition often involves multiple related indexes, which means it can be described in terms of a multiattribute decision-making (MADM) issue that can merely depend on the doctors' experience. Here, Zhang et al. proposed a new set of picture fuzzy point-Choquet integral aggregation operators to resolve the MADM issue [22], which could provide further guidance and direction for enhancing our system.

## 4. Conclusion

The people-oriented integrated delivery system is an effective strategy for coordinating the provision of health services at a lower cost, improving the efficiency and quality of health services, and providing continuous health services. Measurements based on the integrated delivery system can help to improve the healthcare capacity of primary hospitals.

## Figures and Tables

**Figure 1:** Fishbone analysis of problems in primary hospitals.

**Figure 2:** Flowchart of remote consultation.

**Figure 3:** 14 center in Huzhou No. 1 Hospital Medical Group.

**Table 1:** Performance of healthcare in Huzhou No. 1 Hospital before and after taking measures.

	Subject	Scoring criteria	Numerical value		Score	
			Before	After	Before	After
Breadth of diagnosis and treatment	Number of DRG groups in secondary hospitals	Full score will be given to group ≥350, and no score will be given if the score is not reached (full score of 7 points)	348	376	0	7
	Number of township health centers with standard number of outpatient diseases	If the number of diseases is more than or equal to 200 and the year-on-year increase is regarded as reaching the standard (score = full score − number of substandard hospitals *∗* 2, full score of 12 points)	2	6	4	12
	Contracted coverage rate of family doctors in key population	6 points for coverage rate ≥60%, 7 points for 70%, 8 points for 80%, full score for 90%, and no score for less than 60% (full score of 9 points)	79.77%	82.78%	7	8

Efficiency of diagnosis and treatment ability	Average daily diagnosis and treatment times of doctors	No score if it is less than 10, 6 points will be obtained if it is equal to 10, 1 point will be gained for each person who is promoted, and full score will be obtained if the score is greater than or equal to 14 (full score of 10 points)	12	13	8	9
	Bed utilization rate	If it is controlled at 95% ± 2%, 1 point will be deducted for every 3% reduction (full score of 10 points)	83.16%	85.87%	6	7
	Average length of stay	If the average length of stay is less than or equal to 8 days and less than the previous year, full score will be given; otherwise, no score will be given (full score of 10 points)	5.72	5.67	10	10

Surgical ability	Proportion of operations above grade II in secondary hospitals	12 points for more than 30%, 1 point for every 5% increase, full score for more than 70% (full score of 20 points)	56.53%	58.34%	17	17
	Types of operation and therapeutic operation in township hospitals	6 points for more than 30 items, 7 points for 40 items, 8 points for 50 items, 9 points for 60 items, and 10 points for 70 items (full score of 10 points)	32	51	6	8

Patient satisfaction	Outpatient satisfaction	More than 90% get full score, ≥85% score 5 points, ≥75% score 4 points, ≥65% score 3 points, ≥60% score 2 points, less than 60% no score (full score 6 points)	71.32%	88.56%	3	5
	Inpatient satisfaction	More than 90% get full score, ≥85% score 5 points, ≥75% score 4 points, ≥65% score 3 points, ≥60% score 2 points, less than 60% no score (full score 6 points)	70.66%	80.23%	3	4

Total score					**64**	**87**

## Data Availability

The datasets used or analyzed during the current study are available from the corresponding author on reasonable request.
